# Employment of Ensemble Machine Learning Methods for Human Activity Recognition

**DOI:** 10.1155/2022/6963891

**Published:** 2022-09-25

**Authors:** Tasnimul Hasan, Md. Faiyed Bin Karim, Mahin Khan Mahadi, Mirza Muntasir Nishat, Fahim Faisal

**Affiliations:** Department of EEE, Islamic University of Technology, Gazipur, Bangladesh

## Abstract

The endeavor to detect human activities and behaviors is targeted as a real-time detection mechanism that tends to predict the form of human motions and actions. Though sensors like accelerometer and gyroscopes are noticeable in human motion detection, categorizing unique and individual human gestures require software-based assistance. With the widespread implementation of machine learning algorithms, human actions can be distinguished into multiple classes. Several state-of-the-art machine learning algorithms can be applied to this specified field which will give suitable outcomes, yet due to the bulk of the dataset, complexity can be made apparent, which will reduce the efficiency of the model. In our proposed research, ensemble learning methods have been established by assembling several trained and tuned machine learning models. The adopted dataset for the model has been preprocessed through PCA (principal component analysis), SMOTE oversampling (synthetic minority oversampling technique), and K-means clustering, which reduced the dataset to essentials, keeping the weight of the features intact and reducing complexity. Maximum accuracy of 99.36% was achieved from both stacking and voting ensemble methods.

## 1. Introduction

Human activity recognition (HAR) bears significance in human-to-human contact and interpersonal relationships containing identification, personality, and psychological state of people [1]. For instance, when a performer conducts an action figure-focused scene in front of an uncluttered backdrop, the computer can assess and deliver a conclusion, but it appears to be quite challenging because of components that vary in size and frame resolution. However, identifying behavioral roles takes time and requires familiarity with the specific event being reported. In addition, the similarities that occur within and between the courses make the procedure considerably more complex. For example, different people may use distinct body motions to indicate the same kind of action. In spite of this, class actions may be difficult to detect even when they are represented by the same quantity of data. People's habits influence the way they carry out a task, making it harder to discern what they are doing. Another significant problem is to create an actual-time graphic representation for learning and comprehending human behavior with just a few trial results on which to base one's findings [2].

In this context, keeping clients happy in today's fast-paced market relies heavily on technology. Hardware and software upgrades are being introduced into technology to improve performance and efficiency as technology evolves. Many new hardware components are being considered for mobile devices since it is commonly accepted that we cannot do even the simplest task without our smartphones in hand [3]. Moreover, sensors are more important to smartphone designers than other features since they make our lives a little simpler. A growing number of integrated sensors in smartphones are getting smaller and more powerful, allowing them to store a large amount of data from our daily activities that are deemed to be significant [4]. Almost all phones come with an accelerometer as standard equipment. Technological advances in recent years have made it possible to integrate incredible capabilities and a variety of sensors into a single device. This is very astonishing since the vast majority of these devices are found in HAR setups [5]. It is now much simpler to collect and analyze data and transmit data from one place to another, thanks to the growing interaction between hardware and software and sensor gadgets that are doing remarkably well in this fast-moving technological era [6].

Therefore, HAR solutions' success hinges on a grasp of its fundamental concepts, limitations, and problems. Human activities may be seen as a set of recurrent daily acts performed in a certain area across time. If a given action, such as walking or cooking, becomes observable and regular, it may be termed as an activity. Current algorithms to identify human activity have limited predictive power since people do jobs in a variety of ways depending on their own preferences and health as well as habit. High-accuracy sensor data may be utilized to identify the human's everyday activities using machine learning models and deep neural networks, respectively. The accelerometer sensors that are implanted in various places of the body are used to detect movements and identify activities. Each sensor has varying sensitivity to different types of activities [7]. Hence, smartphone usage in HAR is on the rise because of the discomfort of having sensors all over their body as they go about their daily routines.

Machine learning algorithms have emerged as handy tools for developing automated systems in the modern era. For different, classification, detection, prediction, and regression-based analysis, ML algorithms are employed widely by researchers [8–11]. In this paper, sophisticated preprocessing methods [12] have been introduced to minimize dataset size, keeping dataset quality unchanged followed by the employment of several machine learning (ML) algorithms which include Support Vector Classier (SVC), Linear SVC (LSVC), NuSVC, Extreme Gradient Boosting (XGBoost), Adaptive Boosting (Adaboost), Light Gradient Boosting Machine (LGBM), Gradient Boosting (GB), and Extra Trees Classifier (ETC). Moreover, hybrid ensemble machine learning techniques have been implemented, which are defined as stacking, voting, blending, and averaging to train the preprocessed data collected from single and multiple devices. For preprocessing, principal component analysis (PCA) has been brought into action and features have been reduced throughout the process, which has contributed to the reduction of data features as well as in reduction in complexity of training the model. Also, the minority group has been oversampled using SMOTE (synthetic minority oversampling technique), which equaled the amount of each class of samples by increasing the quantity of data. Furthermore, K-means clustering was performed and from elbow plot to silhouette coefficient values, the prominent K-means clustered value was determined. The rest of the paper is arranged as follows: related works and motivation of this study are presented in Section 2. Detailed information on the datasets and methods utilized in the research are depicted in Section 3. And, Section 4 includes the results and discussion of the study followed by the conclusion in Section 5.

## 2. Related Work & Motivation

Many studies have been conducted regarding human activity recognition. For instance, Shakya et al., implemented random forest (RF), decision tree (DT), K-nearest neighbor (KNN), recurrent neural network (RNN), and convolutional neural network (CNN) for identifying human daily activities such as walking and cycling [13]. Among them, CNN displayed the highest accuracy rate of 99.16% in five-fold cross-validation. For balanced datasets, better learning capacity and considerable recognition accuracy with good outcomes were reported. Unbalanced datasets could not produce accurate recognition results. However, Deep and Zheng optimized the detection of human activity using CNN and the long short-term memory (LSTM) technique [14]. This method achieved an accuracy of 93.40%. Significant recognition performance was obtained for an individual's simple and restricted actions. On the other hand, Abbaspour et al. applied four hybrid deep learning models to test performance on the HAR problem using publicly available datasets PAMAP2, where each hybrid model combined a CNN with a range of RNNs, resulting in higher accuracy [15]. The hybrid models employed CNNs with two convolution layers, but the experiment was repeated with CNNs with three and four convolution layers to observe how the number of convolution layers influenced the outcomes. Increasing the number of layers to three and four, on the other hand, resulted in minimal modification in the execution of the GRU-based/LSTM-based models. This model was carried out iteratively to gain better accuracy. In related work, Jaouedi et al. used a mix of the transfer learning model and the RNN model [16]. The features were taken from InceptionV3. Three independent datasets were used to evaluate the model's performance where the model achieved an accuracy of 92%. However, Polu showcased a modified version of a similar ML model on human activity detection [17]. Here, the RF classifier and modified RF classifier were used, where the modified RF classifier gained better performances compared to the conventional RF model. Suto et al. [18] illustrated the difference in performance between online and offline cases of HAR on people of different ages. Among the models, ANN reached the highest recognition rate of 97%. The research also concluded that further improvements were required on the approach for a flawless HAR system as the model had a lack of data expansion problem. A comparative study was observed between the CNN model and other ML models in a similar research by Wan et al. where the CNN model provided superior output compared to the other ML models [19]. Vijayvargiya et al. presented a windowing method for 25% overlapping [20]. Among the models, RF imparted the highest accuracy of 92.71% at 5-fold cross-validation.

For supervised classification methods, the detection of human activities is required to be more precise, time efficient, and more compact when it comes to complexity as the size of the dataset can be bulky and perplexing at times. This study investigates the performances of hybrid ensemble machine learning models with a view to achieve better results from selected hyperparameter-tuned models through a series of actions. Before training the models, the dataset was reduced using principal component analysis (PCA) and was manipulated through SMOTE oversampling and K-means clustering techniques. Thus, the dataset was set off to be more engaging and concise. The hybrid ensemble models namely stacking, voting, blending, and averaging were applied to the tuned ML models which executed the performance more efficiently, producing better performances than the state-of-the-art methods. Application of these hybrid ensemble methods can become a regular practice in the field of a healthcare system where the detection process can be made more functional and user-friendly. Thus, the proposed model can advance in the field of human activity recognition, being capable of making the following contributions:

- Proposing a dimensionality reduction technique of the dataset in preprocessing step where time consumption in simulation is minimized.
- Carrying out a comprehensive investigation of the HAR system by deploying different supervised machine learning algorithms.
- Implementing various ensemble ML models which can demonstrate better detection results of each class among all the designated machine learning models.

The practical administration of the proposed model on real-time human activity detection can significantly facilitate various diagnosis processes in the healthcare system. It can also put an impact on a motion-based road crossing and traffic system as well as observation techniques in the security system. Moreover, the detection process in many other devices and sensors can be mapped in a more sophisticated manner following the implemented model.

## 3. Methodology

### 3.1. Dataset Description

For this study, a thorough exploration was executed and the dataset was finalized for training the models, which is a public domain dataset [21]that is also available on Kaggle [22], one of the most comprehensive and well-known resources [21]. The dataset comprises 10299 occurrences and 561 features. In all, these 10299 cases were categorized into six different categories of activities which were experimented on 30 participants aged between 19 and 48 years. The classification of types for the dataset is listed in Table 1.

An inertial sensor-equipped smartphone was strapped to the waists of 30 study participants as they carried out tasks of daily living. The purpose of this exercise was to identify of a total six actions each participant was performing at any given time. The recordings were then used to compile a HAR database. In order to record 3-axial linear acceleration and 3-axial angular velocity at a steady 50 Hz using an accelerometer and gyroscope that were worn by the participants, a group of 30 willing participants ranging in age from 19 to 48 years old participated in six exercises while wearing the Samsung Galaxy S II around their waists: walking, walking upstairs, walking downstairs, sitting, standing, and lying down. The tests have been videotaped and the resultant dataset was randomly divided into two sets, with 70% of the volunteers contributing to the training data and 30% contributing to the test data accordingly, for the purpose of manually labeling the data. Data were captured using fixed-width sliding windows with a length of 2.56 seconds and an overlap of 50% after noise filters were applied to sensor signals (accelerometer and gyroscope, 128 readings per window). The sensor acceleration data were split up into several categories using a Butterworth lowpass filter to remove the gravitational and body motion components. Because the gravitational force is thought to only be composed of low-frequency components, a filter with a cutoff frequency of 0.3 Hz was used to separate the two categories of body acceleration and gravity. Each window was used to generate a feature vector by completing computations using variables in the time domain and the frequency domain. Each entry in the collection has details about total acceleration and angular velocity obtained from the gyroscope, 561-feature vector with time and frequency domain variables, activity level, and subject identifier.

### 3.2. Data Preprocessing

#### 3.2.1. Min-Max Scaler

A dataset is recommended to be mitigated before training the model with that dataset to reduce training complexity and computational time without decreasing the characteristic depth. A course of actions were taken in order to preprocess the dataset for our approach. At first, the Min-Max scaler was implemented on the selected dataset. The Min-Max scaler is applied on the dataset to standardize the variables and scale them between 0 and 1. The fit transform function is generally used to transform the dataset after it has been defined. Scaling the numbers to a given range without altering the form of the original pattern is what this does.

#### 3.2.2. PCA Method

As the values were scaled, principal component analysis (PCA) was then applied to the dataset [23]. PCA is considered an unsupervised learning strategy to reduce the number of interrelated variables in a dataset, while still providing an accurate assessment by maintaining maximum variance in the data. In our model, it has been applied when dealing with data that have linear correlations but have been plagued by the curse of dimensionality, namely when the presence of too many features leads to noise. This is exacerbated in particular by features with varying scales. While keeping as much variance as possible, PCA's major goal is to minimize the number of dimensions of a dataset composed of a large number of closely related variables. To get PCA to work properly, firstly data are normalized which is accomplished by subtracting the respective means from the values in the relevant column which will provide a 2 × 2 covariance matrix since the dataset is two-dimensional. Then, the covariance matrix, eigenvectors, and eigenvalues are calculated. In order to get the components in order of importance, the eigenvalues from greatest to lowest are sorted where the dimensionality got reduced. There are “*n*” eigenvalues and eigenvectors for every “*n*” variable in a dataset. As it turns out, the most significant eigenvector in the dataset is the eigenvector with the highest eigenvalue. The first few eigenvalues are taken and the remainder is discarded in order to shrink the dimensionality. A minimal number of eigenvalues are enough to ensure not to lose much information in the process. A simultaneous workflow of the PCA method is illustrated in Figure 1.

A feature vector is then constructed by multiplying the eigenvectors by a matrix. Only the eigenvectors are required to continue being included in this list. It is possible to either choose the dimension with the bigger eigenvalue or just take both dimensions. In this last step, everything the arithmetic that has been performed up to this point is used to construct the principal components. When transposing a feature vector, a left-multiply operation is implemented to combine it with a transpose of the original dataset.

At the beginning of the process, standardization is performed on each feature in the dataset which tends to achieve the mean and variance 1 [24]. After that, the covariance matrix of the dataset is formed by computing the covariance [25]. From the covariance matrix, the eigenvectors along with their eigenvalues are measured [26]. Eigenvalues are later on sorted from highest to lowest. From the vectors, top components are selected as features. After applying PCA in our dataset, a graph has been plotted displaying variance with respect to the number of components which is represented in Figure 2. From the PCA method, 120 features were nominated from 561 features.

#### 3.2.3. SMOTE-ENN Technique

Observing the graph, it is visible that, the variance curve is increased to the maximum from the 120 components and after that, the change of variance was not significant as the number of features increased. Reducing the number of features helps in the exploratory data analysis phase, which feeds into the data wrangling phase and model training phase. Next, on the selected 120 features, an oversampling strategy known as synthetic minority oversampling technique (SMOTE) followed by data percentage was performed in which the samples were created for the minority group [27]. With random oversampling, there is a risk of overfitting. So, this method can be performed through either of the four ways fusion of new data from minority class, minority class oversampling, majority class undersampling, and assembling misclassification of minority instances to be more important than misclassification of majority class data through modification of the cost function. Instead of using replacements to oversample, the SMOTE oversampling method generates new synthetics from scratch. In order to oversample samples from the minority class, SMOTE uses synthetic examples in the line segments. It brings together the members of the *K* minority who live in close proximity to one another. The “*k*” closest neighbors' neighbors are chosen at random. According to the quantity of oversampling required, the number is determined.

SMOTE-ENN sampling method is a complete approach that combines the SMOTE and Wilson's Edited Nearest Neighbor Rule sample techniques (ENN). SMOTE is an oversampling approach, and its primary goal is to generate new minority class instances by interpolating between multiple different minority class examples that reside in close proximity to one another, even while it has the potential to significantly increase the model's classification accuracy, it also has the capability of producing noise samples and boundary samples. ENN is a technique that is used as a data cleaning tool that may delete any example whose class label is different from the class of at least two of its three closest neighbors so that better-defined class clusters can be created using ENN. The likelihood of overfitting caused by synthetic examples is decreased by the use of SMOTE-ENN due to the fact that certain instances from the majority class may invade the area reserved for the minority class and vice versa. Because of the ease with which it may be implemented and the high classification performance it offers, the KNN technique is one of the most used classification methods used in the data mining and statistics. The concept behind this is that a sample belongs to a certain category if the majority of the “*k*” samples that are most similar to it, also belong to that category, with “*k*” typically not exceeding 20 in most cases. When using the KNN technique, the objects that are considered to be “neighbors” are those that have successfully been categorized. This approach only uses the category of the sample or samples that are geographically closest to the one that has to be categorized in order to identify which category the sample in question belongs to. The workflow diagram of SMOTE-ENN is presented in Figure 3.

Dup size and *K* are SMOTE's two parameters where the algorithm will examine the viewpoint of current instances and randomly create new ones. The function will generate a new instance at a certain distance from the nearest instance. At *K* = 1, the function will examine the nearest neighbor. At *K* = 2, the function will examine the nearest and subsequent neighbors. Typically, SMOTE algorithm will iterate over the first minority instance. While loop iteration is a single instance, the model creates a new instance between the initial instance and its neighbor. The dup size option specifies the number of times the original instance will be duplicated by the SMOTE function. At dup size = 1, for instance, the model will generate just four additional data points, and so on. Throughout the process, the dataset was leveled to 1944 samples for each class, fabricating it into a dataset of a total of 11664 samples.

#### 3.2.4. K-Means Clustering

After forming the increased data by SMOTE oversampling, K-means clustering has been applied. These are data that are an unsupervised machine learning approach, capable of clustering unlabeled data based on similarities into a preset number of groups [28]. In the case of unlabeled data, the K-means clustering algorithm can be utilized (i.e., data without defined categories or groups). In this method, the number of groups is represented by the variable *K*, which is the purpose of this algorithm. Iteratively assigning each data point to one of the *K* groups is how the method works. Clustering is based on the similarity of the features of the data points. The method divides the data into a number of clusters determined by *K* and obtains a *K* number of the centroid for each cluster. Utilizing these centroids, the closest data points are assigned for each centroid, resulting in a new cluster and calculating variance. The whole process is repeated until there is no new centroid left to be reassigned closest to each data point. Thus, the K-means clustering was performed and Elbow plotting and silhouette scores for different values of *K* were established to crosscheck the best output for the value of K represented in Figures 4 and 5(a)–5(c).

From the elbow plot, it can be observed that, the highest slope is generated when *K* = 2. Again, from silhouette analysis, it can be scrutinized that, the silhouette score is highest at *K* = 2, which is 0.491. Thus, from *K* = 2 clusterings, 121 features were put to use. As the dataset was preprocessed, it was then split into an 80 : 20 train test ratio following stratified train test split. Finally, the dataset was organized for training our targeted machine learning models.

### 3.3. Training Models

#### 3.3.1. Supervised ML Models

Learning a function that maps an input to output is the objective of the machine learning task known as supervised machine learning which requires the use of sample input-output pairs that does the job by drawing conclusions about a function based on labeled training data, which consist of a collection of training instances. In supervised learning, each example is a pair consisting of an input object and the desired output value where input objects are used to train the system to produce the intended output value, and the training data are analyzed by a supervised learning algorithm, which then provides an output that is utilized for mapping additional instances. In this study, at first, several ML models such as SVC [29], NuSVC [30], Linear SVC (LSVC) [31], Adaboost (AdB) [32], XGBoost (XGB) [33], Gradient Boosting (GB) [34], Light GBM (LGBM) [35], and Extra Trees Classifier (ETC) [36] have been implemented with a view to observe the performance parameters.

#### 3.3.2. Ensemble Learning Models

After deploying supervised learning ML models, hybrid ML models (ensemble learning techniques) are employed where concepts like stacking, voting, blending, and averaging are implemented. In the following, the methods are explained in brief:

- Stacking:
- Stacking is the process by which an algorithm learns how to combine the output predictions of submodels to get a more accurate output prediction [37]. The stacking method, which employs two-layer estimators, is used to develop classification and regression models for classification and regression issues. This approach divides the training data into two subsets: training and holdout. As a result of stratified sampling with replacement, different learning algorithms create *n* classifiers. The technique is comprises SVC, LSVC, NuSVC, XGB, LGBM, and ETC to create a weight distribution vector for the meta classifier. The workflow diagram of the stacking ensemble model is depicted in Figure 6.
- Voting:
- The voting classifier in machine learning uses an ensemble of multiple models to forecast an output (class) based on the chance that the result will fall into one of the specified classes [38]. Using the most popular class as a starting point, this classifier predicts the output class based on an average of all the classifiers that have been submitted to it. For each output class, a single model might be constructed that trains on several models and predict output based on the aggregate majority of votes for each class. Classification issues are often solved using the maximum voting approach. Multiple models are employed to forecast the outcome of each data point in this method. Using each model's predictions as a vote, we can see how the results differ. Hard voting has been employed in our model using SVC, LSVC, NuSVC, XGB, and LGBM classifiers where the final forecast was based on the results of the majority of the models. The workflow diagram of the voting classifier is illustrated in Figure 7.
- Blending:
- Blending is an approach in ensemble machine learning that makes use of a machine learning model that learns the best effective way to combine the predictions from various contributing ensemble member models [39]. When it comes to making predictions, blending is similar to stacking in that, it only uses a holdout (validation) set from the train set. To put it another way, predictions are only made on the holdout set, rather than on the whole set of forecasts. When the holdout set and predictions are combined, a model is formed, and the model is then evaluated on the test set. As a first step, the dataset is separated into two sections, the training set and the testing set. Following that, the train set is divided into two parts: the training set and the validation set. As for our implementation of the blending model LSVC, NuSVC, LGBM, XGB, and ETC are fitted to the training set while predictions are produced based on the validation set and the test set, respectively. The validation set and its predictions are utilized as features in the construction of a new model, which is designated as SVC. In order to create final predictions about the test set with its produced meta-features, this model is utilized. The basic working principle of the blending method is presented in pictorial form in Figure 8.
- Averaging:
- In averaging, numerous forecasts are created for each data point, in a manner similar to the maximum voting strategy [40]. In this procedure, an average of the predictions is taken from all of the models and is used to generate the final prediction. Averaging can be used to make predictions in regression problems, as well as to calculate probabilities in classification issues, among other applications. The algorithms such as SVC, NuSVC, LGBM, and XGB were combined in the averaging model to observe performance and make the final prediction. The averaging technique is illustrated in Figure 9.

To sum up the whole process, the elected dataset was firstly preprocessed with PCA, SMOTE, K Means clustering, elbow method, and Silhouette analysis accordingly. Afterward, the data were split into test data and train data, which later on was utilized to train the machine learning models with hyperparameter tuning enhanced. Also, mentioned hybrid ML models were generated and trained by the dataset, which gave a more efficient outcome. The whole workflow diagram for our proposed model is illustrated in Figure 10.

## 4. Result & Analysis

After processing the dataset, the ML models were trained and the results are presented. For achieving better results, hyperparameters are tuned. Instead of using other parameters, hyperparameters are used because they are able to handle the number of polynomial features that should be used in the linear model, the maximum decision tree depth that is permitted in the decision tree, the number of samples that should be used at each leaf node, and the optimal number of layers for the network. Parameter values that were set for the hyperparameter tuning on the ML models are indexed in Table 2.

The performances of the trained models in both “tuned” and “without tuned” were assessed by employing rigorous simulation in Python. Performances of the individual models were tweaked through hyperparameter tuning and with the tuned models, a hybrid model was established. For a given set of test data, the confusion matrix is a matrix used to evaluate the performance of classification models. Test data values can only be determined if they are known. Predicted and actual values, as well as the total number of predicted values, may be found in two dimensions of the matrix. In the context of a model, predicted values are those values that the model predicts, and actual values are those values that the model actually predicts based on the observed data. As a result, it shows us how well the classification model performs in terms of making predictions on test data. It reveals not only the kind of mistake produced by the classifiers but also the number of errors they made. Each algorithm's accuracy, precision, F-score, and recall are computed using the confusion matrix as a source. The confusion matrices indicate not just the outputs of predictive models, but rather which classes are properly predicted, which are erroneously forecasted, and what sorts of issues are forming. The evaluation matrices obtained through training the ML models are represented from Figures 11–30.

As the confusion matrices were produced, classification efficiency was comprehensible from the output. Thus, several performance metrics were evaluated which are defined as accuracy, micro precision, macro precision, weighted precision, micro recall, macro recall, weighted recall, micro *F*1-score, macro *F*1-score, weighted *F*1-score, and cross-validation score. Accuracy is defined as the percentage of total correctly predicted values among all predicted values. Also, the precision of an ML model indicates the efficiency of detecting true positive values among all correctly predicted values whereas recall demonstrates the number of correctly identified true positive values among total predicted values of a specific class. Finally, *F*1-score is produced from precision and recall, which is the weighted average of these two parameters.

For measuring micro values

(1) $$\begin{array}{c} Accuracy=\frac{TP+TN}{TP+TN+FP+FN}\text{,}\\ Micro\;Precision=\frac{total\;TP}{total\;TP+total\;FP}\text{,}\\ Micro\;Recall=\frac{total\;TP}{total\;TP+total\;FN}\text{,}\\ Micro\;F1-score=2\times \frac{Micro\;Precision\times Micro\;Recall}{Micro\;Precision+Micro\;Recall}. \end{array}$$

For calculating macro and weighted values

(2) $$\begin{array}{c} Precision=\frac{TP}{TP+FP},\\ Recall=\frac{TP}{TP+FN},\\ F1-score=2\times \frac{Precision\times Recall}{Precision+Recall},\\ Macro\;Precision=\frac{\sum_{k=0}^{n}Precision_{k}}{n},\\ Macro\;Recall=\frac{\sum_{k=0}^{n}Recall_{k}}{n},\\ Macro\;F1=\frac{\sum_{k=0}^{n}F1-score_{k}}{n},\\ Weighte\;d\;Precision=\frac{\sum_{k=0}^{n}\left(Precision_{k}\times True\;value_{k}\right)}{\sum_{k=0}^{n}True\;value_{k}},\\ Weighte\;d\;Recall=\frac{\sum_{k=0}^{n}\left(Recall_{k}\times True\;value_{k}\right)}{\sum_{k=0}^{n}True\;value_{k}},\\ Weighte\;d\;F1=\frac{\sum_{k=0}^{n}\left(F1-score_{k}\times True\;value_{k}\right)}{\sum_{k=0}^{n}True\;value_{k}}. \end{array}$$

After observing and applying relevant equations on the confusion matrices of trained ML models, the required performance parameters were obtained. Performance metrics of the machine learning models are tabulated in Tables 3 and 4 representing models trained without hyperparameter tuned and with hyperparameter tuned states, accordingly.  Table 5 presents the results obtained from trained hybrid models.

As the models were initially trained and performances of such were visualized in Table 3, it is observed that SVC attained the highest accuracy of 98.37% among all the models, surpassing the accuracy of LSVC which was 98.87%. Moreover, SVC outperformed other ML models in other performance metrics too, obtaining the precision value of 0.9837 (micro, macro, and weighted), recall of 0.9837 (micro, macro, and weighted), and *F*1-score of 0.9837. But, in the case of cross-validation score, linear SVC gained the highest score of 0.9701 among all ML models. On the other hand, XGBoost displayed the highest accuracy of 97.64% among all trained boosting algorithms. Conversely, AdaBoost performed with an accuracy of 40.08%, which is reported to achieve the lowest accuracy among all models. In Tables 4 and 5, the performance metrics of hyperparameter tuned ML models and hybrid models were demonstrated respectively. Among all these models, the stacking model and voting model performed most efficiently among all ML models, gaining an accuracy of 99.36%. Aside from the hybrid models, SVC achieved the highest accuracy of 99.31% among all tuned models, leaving behind the averaging model and NuSVC with the accuracies of 99.27% and 99.23% respectively. Also, the blending model achieved an accuracy of 99.1%. On the other hand, among the boosting models, XGBoost gained the highest accuracy of 98.59%. Furthermore, it is observed that after hyperparameter tuning the performances of the ML models improved notably. The most significant development due to hyperparameter tuning was detected on AdaBoost, which had an increased accuracy of 81.95% from 40.08%. In the case of precision, recall, and F1-score (micro, macro, and weighted), stacking and voting models surpassed other ML models, both acquiring a precision value of 0.9936 (micro, macro, and weighted), recall of 0.991 (micro, macro, and weighted), and *F*1-score of 0.9936 (micro, macro, and weighted). Above that, it is also seen that hybrid models exhibit optimum performance in all types of performance metrics compared to the individual state-of-the-art methods even when hyperparameter tuning has been adjusted on the individual training models. To have a broader and thorough idea about the efficiency of the research model, a comparative analysis has been carried out between our research models and the approached classification models of other authors, which classified the dataset of human activities which is similar to ours. A brief comparison has been tabulated in Table 6.

## 5. Conclusion

Human movement acknowledgment, which plans to perceive the practices and goals of at least one specialist in light of a succession of perceptions on the specialists' activities and the encompassing conditions is the establishment for a considerable length of time for instances, video reconnaissance, medical services, and human-computer connection. Human action acknowledgment has several practices in clinical examination and human overview frameworks, but there are snags while managing reasonable scenes, notwithstanding the inborn intraclass fluctuation and interclass likeness issue. Moreover, any human conduct might be promptly appreciated and made a lot simpler by using wise ML-based calculations that can be utilized because of its capability. In this research, a general correlation is made as far as a few presentation factors for effectively recognizing human conduct. The models were trained effectively as the dataset was preprocessed by rigorous and thorough methods of PCA, SMOTE, and K-means clustering, which kept the dataset features compact. Moreover, hybrid models have been utilized from the hyperparameter tuned state-of-the-art methods which demonstrated to be more efficient compared to the individual algorithms as two of the hybrid models obtained the highest accuracy of 99.36%, which are stacking and voting models. As the dataset was preprocessed and efficient hybrid models were introduced, significantly precise and shrewd outcomes were achieved as expected. As a supervised machine learning model, our proposed methods are expected to perform on a larger and bulkier dataset with a consistent outcome that may be utilized practically in the field of activity recognition process on human beings and reduce the complexity and expenses of the recognition process as well.

## Figures and Tables

**Figure 1:** Workflow diagram of the PCA method.

**Figure 2:** Variance through increasing the number of components.

**Figure 3:** The workflow diagram of SMOTE-ENN.

**Figure 4:** Elbow plot on different *K* clustered values applied on sample data.

**Figure 5:** Silhouette analysis for K-means clustering on sample data with (a) *K* = 2, (b) *K* = 3, and (c) *K* = 4.

**Figure 6:** The workflow diagram of stacking ensemble model.

**Figure 7:** The workflow diagram of voting classifier.

**Figure 8:** The basic workflow diagram of blending ensemble model.

**Figure 9:** The workflow diagram of averaging ensemble model.

**Figure 10:** The proposed methodology for human activity recognition.

**Figure 11:** Confusion matrix of SVC (without tuning).

**Figure 12:** Confusion matrix of SVC (with tuning).

**Figure 13:** Confusion matrix of NuSVC (without tuning).

**Figure 14:** Confusion matrix of NuSVC (with tuning).

**Figure 15:** Confusion matrix of linear SVC (without tuning).

**Figure 16:** Confusion matrix of linear SVC (with tuning).

**Figure 17:** Confusion matrix of AdaBoost (without tuning).

**Figure 18:** Confusion matrix of AdaBoost (with tuning).

**Figure 19:** Confusion matrix of gradient boosting (without tuning).

**Figure 20:** Confusion matrix of gradient boosting (with tuning).

**Figure 21:** Confusion matrix of XGBoost (without tuning).

**Figure 22:** Confusion matrix of XGBoost (with tuning).

**Figure 23:** Confusion matrix of LGBM (without tuning).

**Figure 24:** Confusion matrix of LGBM (with tuning).

**Figure 25:** Confusion matrix of extra trees classifier (without tuning).

**Figure 26:** Confusion matrix of extra trees classifier (with tuning).

**Figure 27:** Confusion matrix of the stacking model.

**Figure 28:** Confusion matrix of the voting model.

**Figure 29:** Confusion matrix of the averaging model.

**Figure 30:** Confusion matrix of the blending model.

**Table 1:** Dataset sample types for the proposed model.

No.	Type of activities	Samples
1	Walking	1722
2	Walking upstairs	1544
3	Walking downstairs	1406
4	Sitting	1777
5	Standing	1906
6	Laying	1944

**Table 2:** Hyperparameter tuning values of ML models.

Training model	Parameter	Value
SVC	*C*	10.4

NuSVC	nu	0.0131

LSVC	*C*	20.30

XGB	Learning rate	0.239
	Max depth	6

AdB	Learning rate	0.31
	Algorithm	“SAMME.R”
	*n*_estimators	138

LGBM	Boosting_type	“Goss”
	Learning rate	0.51
	*n*_estimators	124
	Num_leaves	31

GB	Learning rate	0.401
	*n*_estimators	85

ETC	*n*_estimators	123

**Table 3:** Performance metrics of trained ML models (without tuning).

Algorithm	Accuracy	Precision (micro)	Precision (macro)	Precision (weighted)	Recall (micro)	Recall (macro)	Recall (weighted)	*F*1-score (micro)	*F*1-score (macro)	*F*1-score (weighted)	Cross-validation score
SVC	0.9837	0.9837	0.9837	0.9837	0.9837	0.9837	0.9837	0.9837	0.9837	0.9837	0.9681
LSVC	0.9816	0.9816	0.9815	0.9815	0.9816	0.9816	0.9816	0.9816	0.9815	0.9815	0.9701
NuSVC	0.9387	0.9387	0.9401	0.9401	0.9387	0.9387	0.9387	0.9387	0.9388	0.9388	0.926
AdB	0.4008	0.4008	0.2864	0.2863	0.401	0.4010	0.4008	0.4008	0.2723	0.2721	0.4049
XGB	0.9764	0.9764	0.9763	0.9763	0.976	0.9764	0.9764	0.9764	0.9763	0.9763	0.9547
LGBM	0.9747	0.9747	0.9746	0.9747	0.975	0.9747	0.9747	0.9747	0.9747	0.9747	0.9475
GB	0.9587	0.9587	0.9600	0.9590	0.9689	0.9699	0.9689	0.9587	0.9597	0.9587	0.9148
ETC	0.9627	0.9627	0.9626	0.9626	0.9597	0.9597	0.9597	0.9627	0.9626	0.9626	0.9395

**Table 4:** Performance metrics of trained ML models (with tuning).

Algorithm	Accuracy	Precision (micro)	Precision (macro)	Precision (weighted)	Recall (micro)	Recall (macro)	Recall (weighted)	*F*1-score (micro)	*F*1-score (macro)	*F*1-score (weighted)	Cross-validation score
SVC	0.9931	0.9931	0.9931	0.9932	0.9931	0.9931	0.9931	0.9931	0.9931	0.9931	0.9775
LSVC	0.9854	0.9854	0.9854	0.9854	0.9854	0.9854	0.9854	0.9854	0.9854	0.9854	0.972
NuSVC	0.9923	0.9923	0.9923	0.9923	0.9923	0.9923	0.9923	0.9923	0.9923	0.9923	0.9793
AdB	0.8195	0.8195	0.8226	0.8227	0.8195	0.8194	0.8196	0.8195	0.8199	0.8200	0.7469
XGB	0.9786	0.9786	0.9785	0.9785	0.9786	0.9786	0.9786	0.9786	0.9785	0.9785	0.9517
LGBM	0.9859	0.9859	0.9858	0.9858	0.9859	0.9859	0.9859	0.9859	0.9858	0.9858	0.9606
GB	0.9689	0.9689	0.9702	0.9691	0.9689	0.9699	0.9689	0.9689	0.9699	0.9689	0.9187
ETC	0.9709	0.9709	0.9709	0.9709	0.9717	0.9717	0.9717	0.9709	0.9707	0.9708	0.9411

**Table 5:** Performance metrics of trained ensemble ML models (with tuning).

Algorithm	Accuracy	Precision (micro)	Precision (macro)	Precision (weighted)	Recall (micro)	Recall (macro)	Recall (weighted)	*F*1-score (micro)	*F*1-score (macro)	*F*1-score (weighted)	Cross-validation score
Stacking	0.9936	0.9936	0.9936	0.9936	0.9936	0.9936	0.9936	0.9936	0.9936	0.9936	0.9793
Voting	0.9936	0.9936	0.9936	0.9936	0.9936	0.9936	0.9936	0.9936	0.9936	0.9936	0.9765
Blending	0.991	0.991	0.9910	0.9910	0.9910	0.9910	0.9910	0.9910	0.991	0.9910	-
Averaging	0.9927	0.9927	0.9927	0.9927	0.9927	0.9927	0.9927	0.9927	0.9927	0.9927	-

**Table 6:** Comparison with other approached models.

Authors	Best trained model	Highest accuracy (%)
Shakya et al. [13]	CNN	99.16
Deep and Zheng [14]	CNN-LSTM	93.40
Jaouedi et al. [16]	RNN	92.00
Polu [17]	Modified RF classifier	94.00
Suto et al. [18]	ANN	97.00
Wan et al. [19]	CNN	92.71
Vijayvargiya et al. [20]	Random forest classifier	92.71
Our research approach	Stacking and voting	99.36

## Data Availability

Human Activity Recognition with Smartphones: Dataset from Kaggle was used in order to support this study and is available at “https://www.kaggle.com/datasets/uciml/human-activity-recognition-with-smartphones”. The dataset is cited at relevant places within the text as Ref [22].

## References

[1] Ramasamy Ramamurthy S., Roy N. (2018). Recent trends in machine learning for human activity recognition—a survey. *Wiley Interdisciplinary Reviews: Data Mining and Knowledge Discovery*.

[2] Arac A., Zhao P., Dobkin B. H., Carmichael S. T., Golshani P. (2019). DeepBehavior: a deep learning toolbox for automated analysis of animal and human behavior imaging data. *Frontiers in Systems Neuroscience*.

[3] De Reuver M., Nikou S., Bouwman H. (2016). Domestication of smartphones and mobile applications: a quantitative mixed-method study. *Mobile Media & Communication*.

[4] Wang Y., Chen Y. J., Yang J. (2016). Determining driver phone use by exploiting smartphone integrated sensors. *IEEE Transactions on Mobile Computing*.

[5] Ramanujam E., Perumal T., Padmavathi S. (2021). Human activity recognition with smartphone and wearable sensors using deep learning techniques: a review. *IEEE Sensors Journal*.

[6] Tran D. N., Phan D. D. Human activities recognition in android smartphone using support vector machine.

[7] Bødker S. (2021). *Through the Interface: A Human Activity Approach to User Interface Design*.

[8] Asif M., Nishat M., Faisal F., Dip R. R. (2021). Performance evaluation and comparative analysis of different machine learning algorithms in predicting cardiovascular disease. *Engineering Letters*.

[9] Nishat M. M., Faisal F., Dip R. (2018). A comprehensive analysis on detecting chronic kidney disease by employing machine learning algorithms. *EAI Endorsed Transactions on Pervasive Health and Technology*.

[10] Nishat M. M., Faisal F., Ratul I. J. (2022). A Comprehensive Investigation of the Performances of Different Machine Learning Classifiers with SMOTE-ENN Oversampling Technique and Hyperparameter Optimization for Imbalanced Heart Failure Dataset. *Scientific Programming*.

[11] Rajput D. S., Basha S. M., Xin Q. (2022). Providing diagnosis on diabetes using cloud computing environment to the people living in rural areas of India. *Journal of Ambient Intelligence and Humanized Computing*.

[12] Misra P., Arun S. Y. Impact of preprocessing methods on healthcare predictions.

[13] Shakya S. R., Zhang C., Zhou Z. (2018). Comparative study of machine learning and deep learning architecture for human activity recognition using accelerometer data. *Int. J. Mach. Learn. Comput*.

[14] Deep S., Zheng X. Hybrid model featuring CNN and LSTM architecture for human activity recognition on smartphone sensor data.

[15] Abbaspour S., Fotouhi F., Sedaghatbaf A., Fotouhi H., Vahabi M., Linden M. (2020). A comparative analysis of hybrid deep learning models for human activity recognition. *Sensors*.

[16] Jaouedi N., Boujnah N., Bouhlel M. (2021). A novel recurrent neural networks architecture for behavior analysis. *The International Arab Journal of Information Technology*.

[17] Polu S. K. (2018). Human activity recognition on smartphones using machine learning algorithms. *International Journal for Innovative Research in Science & Technology*.

[18] Suto J., Oniga S., Lung C., Orha I. (2018). Comparison of offline and real-time human activity recognition results using machine learning techniques. *Neural Computing and Applications*.

[19] Wan S., Qi L., Xu X., Tong C., Gu Z. (2020). Deep learning models for real-time human activity recognition with smartphones. *Mobile Networks and Applications*.

[20] Vijayvargiya A., Kumari N., Gupta P., Kumar R. Implementation of machine learning algorithms for human activity recognition.

[21] Anguita D., Ghio A., Oneto L., Parra X., Jorge L., Reyes-Ortiz A Public Domain Dataset for Human Activity Recognition Using Smartphones.

[22] Kaggle Human activity recognition with samrtphones. https://www.kaggle.com/uciml/human-activity-recognition-with-smartphones/activity.

[23] Anupama Y. K., Amutha S., Ramesh Babu D. R. Exploring efficient preprocessing techniques for breast cancer diagnosis.

[24] Hegde V., Shilpa M., Pallavi M. S. Extracting attributes of students mental health, behaviour, attendance and performance in academics during COVID-19 pandemic using PCA technique.

[25] Misawa K. (2022). Relationships among evolutionary distance, the variance–covariance matrix, multidimensional scaling, and principal component analysis.

[26] Fernandes R., Furtado S. (2022). Efficiency of the principal eigenvector of some triple perturbed consistent matrices. *European Journal of Operational Research*.

[27] Amirruddin A. D., Muharam F. M., Ismail M. H., Tan N. P., Ismail M. F. (2022). Synthetic Minority Over-sampling TEchnique (SMOTE) and Logistic Model Tree (LMT)-Adaptive Boosting algorithms for classifying imbalanced datasets of nutrient and chlorophyll sufficiency levels of oil palm (Elaeis guineensis) using spectroradiometers and unmanned aerial vehicles. *Computers and Electronics in Agriculture*.

[28] Ghazal T. M., Hussain M. Z., Raed A. (2021). Said, afrozah nadeem, mohammad kamrul hasan, munir ahmad, muhammad adnan khan, and muhammad tahir naseem. *Performances of K-Means Clustering Algorithm with Different Distance Metrics*.

[29] Nishat M. M., Faisal F., Hasan T., Karim M. F. B., Islam Z., Shagor M. R. K. An investigative approach to employ support vector classifier as a potential detector of brain cancer from MRI dataset.

[30] Bhat S., Mehbodniya A., Elsayed A., Webber J., Al-Begain K. (2021). Human recognition using single-input-single-output channel model and support vector machines. *International Journal of Advanced Computer Science and Applications*.

[31] Kong W., He L., Wang H. Exploratory data analysis of human activity recognition based on smart phone. *IEEE Access*.

[32] Subasi A., Dammas D. H., Alghamdi R. D. (2018). Sensor based human activity recognition using adaboost ensemble classifier. *Procedia Computer Science*.

[33] Indumathi V., Prabakeran S. A comparative analysis on sensor-based human activity recognition using various deep learning techniques.

[34] Sekiguchi R., Abe K., Yokoyama T., Kumano M., Kawakatsu M. Ensemble learning for human activity recognition.

[35] Csizmadia G., Liszkai-Peres K., Ferdinandy B., Miklósi Á., Konok V. (2021). Human Activity Recognition of Children with Wearable Devices Using LightGBM Machine Learning. *Scientific Reports*.

[36] Uddin Md T., Uddiny Md A. Human activity recognition from wearable sensors using extremely randomized trees.

[37] Gupta A., Jain V., Singh A. (2021). Stacking ensemble-based intelligent machine learning model for predicting post-COVID-19 complications. *New Generation Computing*.

[38] Peppes N., Daskalakis E., Alexakis T., Adamopoulou E., Demestichas K. (2021). Performance of machine learning-based multi-model voting ensemble methods for network threat detection in agriculture 4.0. *Sensors*.

[39] Shukla H., Jagtap N., Patil B. Enhanced Twitter bot detection using ensemble machine learning.

[40] Abba S. I., Linh N. T. T., Abdullahi J. (2020). Hybrid machine learning ensemble techniques for modeling dissolved oxygen concentration. *IEEE Access*.

